The article "Regulation of circGOLPH3 and its binding protein CBX7 on the proliferation and apoptosis of prostate cancer cells" was retracted in 2024. Reasons: duplicated images; overlap with earlier publications.

# Regulation of circGOLPH3 and its binding protein CBX7 on the proliferation and apoptosis of prostate cancer cells

**DOI:** 10.1042/BSR20200936

**Published:** 2020-12-14

**Authors:** Lifeng Gong, Yu Tang, Li Jiang, Wei Tang, Shengjun Luo

**Affiliations:** 1 Chengdu Second People's Hospital, Chengdu 10017, P.R. China; 2 Department of Urology, The First Affiliated Hospital of Chongqing Medical University, Chongqing, 400010, P.R. China

**Keywords:** apoptosis, CBX7, cell proliferation, circGOLPH3, prostate cancer

## Abstract

To clarify the mechanism of circGOLPH3 regulation on prostate cancer cells, we performed an overexpression and interference circGOLPH3 assay in prostate cancer cells PC-3 and then evaluated cellular viability, proliferation, cell cycle, and apoptosis of prostate cancer cells by MTT, CCK8, Edu stain, TUNEL stain, and flow cytometry. Binding proteins of CircGOLPH3 were identified by RNA pull-down, mass spectrometry, and RNA-binding protein immunoprecipitation (RIP) assays. The expressions of CircGOLPH3 and CBX7 were measured by qRT-PCR. The results showed that after overexpression of circGOLPH3, the proliferative capacity and the viability of PC-3cells were significantly improved, whereas apoptosis was inhibited. CircGOLPH3 could bind to the CBX7 protein that was highly expressed in the PC-3 cell. Additionally, a functional test on CBX7 showed that the CBX7 overexpression notably improved the proliferative capacity and the viability of PC-3 cells and decreased cellular apoptosis, which was consistent with the effects of circGOLPH3. The validated the present study that circGOLPH3 and its binding protein CBX7 can promote prostate cancer cell proliferation and inhibit apoptosis.

## Introduction

CircRNA is a natural type of endogenous RNA that reversely splices through gene transcription and post-transcriptional regulation, participating in various cellular physiology and disease processes [1]. They were first found in viruses and thought to be derived from mis-splicing of gene sequences. In recent years, with the development of high-throughput sequencing and bioinformatics analysis, more circRNAs have been unveiled in multitudinous organisms including bacteria, plants, and animals. CircRNA is evolutionarily conserved, stable, and more abundant in exosomes. Although it is considered as a new type of ncRNA, several studies have verified that some circRNAs can translate proteins. More importantly, circRNAs’ expression patterns are tissue-specific and cell-specific. This implies that circRNA holds important biological functions and can be served to diagnose and cure certain diseases as well as cancers. So, albeit little we know the biological functions of circRNA, some circRNAs have been still proved to be associated with diabetes, myocardial infarction, osteoarthritis, Alzheimer’s disease, and even cancers. Previous studies showed that a variety of circRNAs play an important role in esophageal cell carcinoma, liver cancer, gastric cancer, colon cancer, bladder cancer, ovarian cancer, and pancreatic duct adenocarcinoma [2,3]. Prostate cancer is the most common malignant tumor in male reproductive system, and it is the second most common cause of male death. More and more studies showed that an abnormal expression of ncRNA might lead to excessive proliferation, metastasis, and drug resistance of prostate cancer cells. PCA3, PCAT-1, MALAT1, miR-205, miR-34a, and even many other ncRNAs have been reported to be involved in the onset and progression of prostate cancer, and they can be used as potential biomarkers and therapeutic targets for prostate cancer [4,5].

Previous studies pointed out that the circGOLPH3 expression in prostate cancer was obviously higher than the normal prostate tissue [6]. And the data from TCGA database show that the circGOLPH3 level in prostate cancer is the highest among all kinds of cancers. Our study was to investigate the function of circGOLPH3 in prostate cancer and its molecular regulatory mechanism. We overexpressed circGOLPH3 in the PC-3 cell lines and determined its effects on PC-3 cell cycle, proliferation, and apoptosis. CircGOLPH3 binding protein was screened by pulldown and mass spectrometry, whose function was then verified. And all studies above clarified the regulatory functions of circGOLPH3 and its binding protein in prostate cancer.

## Materials and methods

### Cells and cell culture

Prostate cancer (PCa) cell lines PC-3 and nontumorigenic human prostatic epithelial cell line (RWPE-1) were purchased from American Type Culture Collection (ATCC). PC-3 was cultivated with Roswell Park Memorial Institute (RPMI) 1640 medium containing 10% fetal bovine serum (FBS) and 1% penicillin/streptomycin; RWPE-1 was cultured in prostate epithelial cell medium containing 10% FBS and 1% penicillin/streptomycin; all the cells were cultured in a 5% CO_2_ humidified incubator at 37°C.

### Cell transfection

siRNA-circGOLPH3, overexpression (OE)-circGOLPH3, empty vector-circGOLPH3 (OE-NC), OE-CBX7, empty vector-CBX7, si-CBX7, and siRNA negative control (si-NC, Cat. #4390843) plasmids were synthesized and constructed by Shanghai Gemma Biotechnology. Retroviral vectors pGPU/Hygro was utilized to express CBX7. The linearized circGOLPH3 sequences (hsa_circ_0072068) was cloned into the Lentivirus overexpression vector pLC5-ciR. siRNAs transfection was carried with Lipofectamine RNAiMax reagent (ThermoFisher). Cells were seeded in 6-well plates at 3 × 10^5^/well and transfected at the next day with the transfection mixture (9 ml lipofectamine RNAiMax and 30 pmol siRNAs in Opti-MEM I Reduced Serum Medium (ThermoFisher)); there was at least 24-h culture before cell collection and subsequent experiments. PC-3 cells were transfected with OE-circGOLPH3, OE-CBX7, or their empty vector by Lipofectamine 3000 (ThermoFisher) separately following the manufacturer’s protocol. The transfected cells were harvested in 24 h after transfection for RNA extraction or downstream assays. The targeting sequences (5′-3′) were shown as follows: siRNA-circGOLPH3, TTACACATCATTTCTCGAGAA; OE-CBX7, F-ATGGAGCTGTCAGCCATCG, R-TCAGAACTTCCCACTGCGGTC; si-CBX7, AACCACCTGCCTATCTCTTAA.

### Immunofluorescence detection

PC-3 cells were inoculated on 24-well plates for 24 h. Cells were fixed with 4% paraformaldehyde for 15 min, slides were washed three times with PBS for 3 min each time; 5% BSA was added for immersion of 30 min; the blocking solution was aspirated, primary antibody (1:200, Abcam, U.K.) was added for overnight incubation at 4°C. Primary antibody CD133 (ab216323), CD44 (ab189524) and Integrin alpha2beta1 (ab30483) were purchased from Abcam. The slides were washed three times with PBST for 3 min each time. The secondary antibody Goat anti-Rat IgG H&L (1:1000, ab150160, Abcam, U.K.) was added, and the incubation was carried out for 1 h at 37°C. The slides were washed three times with PBST for 3 min each time; the DAPI was added, and the incubation was carried out for 10 min in the dark and washed three times with PBST for 5 min each time; Fluorescence was observed under a fluorescence microscope (Olympus, Japan). Red represents positive cells.

### EdU stain assay

PC-3 cells were incubated in DMEM medium containing 10 mM EdU for 24 h. After incubation, the cells were fixed with 4% paraformaldehyde for 30 min and then neutralised with 2 mg/ml glycine for 5 min. Cells were washed three times with PBST for 10 min. Cells were then stained by Apollo and Hoechst33342.

### TUNEL stain assay

Cells were fixed with 4% paraformaldehyde for 20 min at room temperature. Cells were stained according to the manufacturer’s instructions of the TUNEL Kit [cat. no. 11684817910; Roche Diagnostics (Shanghai) Co., Ltd.]. The apoptotic cell was observed at a magnification of ×100 using an inverted fluorescence microscope (cat. no. CKX53; Olympus Corporation), with red representing apoptotic cells and blue representing the nucleus pulposus.

### MTT detection

Every single cell suspension was prepared with a culture solution of 10% fetal calf serum, within which prostate cancer cells were cultured. The cells were seeded into a 96-well plate in a density of 1000–10,000 cells per well, and the volume of each well was 200 μl. The cells are cultured under the same general conditions for 3–5 days (the culture time can be determined according to the test purpose and requirements). After 3–5 days of coloration, 20 μl of MTT solution (5 mg/ml in PBS) was added to each well. The cell culture was lasted for 4 h and then terminated. Carefully aspirate the culture supernatant of each well. After that, the culture supernatant from wells was further centrifuged and then aspirated to suspend the cells. Add 150 μl DMSO to each well and shake the plate for 10 min to fully dissolve the crystals. The wavelength for colorimetry was determined at 490 nm, the light absorption value of each well was measured on the enzyme-linked immunosorbent monitor then the results were recorded, and the cell growth curve was drawn.

### CCK8 proliferation experiment

Cell suspensions (100 μl/well) were seeded in 96-well plates. And the culture plates were kept in the incubator for pre-culture (37°C, 5% CO_2_). After treatment, 10 μl of CCK solution was added to each well (be careful not to generate air bubbles in the wells, they will affect the reading of the OD value). The culture plates were kept in an incubator for 1–4 h. The absorbance at 450 nm was measured with microplate reader.

If the OD value wouldn’t be measured immediately, 10 μl of a 0.1 M HCl solution or a 1% w/v SDS solution was added to each well, and the culture plates were covered with a culture plate and stored under room temperature in a dark place. There won’t be any change when the measurement was performed within 24 h.

### Flow cytometry for cell cycle

Prostate cancer cells in the growth phase were washed with PBS, and then treated with 1 ml trypsin for 1–5 min. Cell suspensions of 5 ml PBS were prepared and then transferred into 15 ml centrifuge tubes, centrifuged at 1500 rpm for 5 min; whose supernatant was removed. Another 500 μl of PBS was added, and the cell pellets were gently blown away into a cell suspension, then 2 ml of 20°C 95% cold ethanol dropwise was added in a vortex state; 30 min of standing for well-mixing and fixing.

Addition of 5 ml PBS was then added into the tube, which was centrifuged at 1500 rpm for 5 min; the supernatant was discarded. About 5 ml PBS was added to resuspend the cells, which was centrifuged at 1500 rpm for 5 min, then the supernatant was removed. About 800 μl PI staining solution was utilized to blow the cell pellet away and to mix it well, being stained at room temperature for 30 min in the dark. Flow cytometry was subsequently performed.

### Flow cytometry for apoptosis experiment

Prostate cancer cells were directly collected into a 10 ml of centrifuge tube. The number of cells in each sample was (1–5) × 106/ml, centrifuged at 1000 r/min for 5 min, and the culture solution was discarded. The cells were washed once with incubation buffer and centrifuged at 1000 r/min for 5 min. Resuspend it with 100 μl of the labeling solution and incubate it at room temperature for 10–15 min in the dark. After that, the samples were centrifuged at 1000 r/min for 5 min and the pellets were washed with incubation buffer once. Then the samples were incubated with fluorescent (SA-FLOUS) solution at 4°C for 20 min in dark, shaken occasionally. Flow cytometer excitation light wavelength was determined at 488 nm. FITC fluorescence was detected with a passband filter with a wavelength of 515 nm, and PI was detected with a filter with a wavelength greater than 560 nm.

### *In vitro* transcription and RNA pulldown

Prepare the reaction system according to the following ratio: 1 μl 10× Transcription Buffer (Ambion); 1 μl 10× NTPs (4 mM ATP, CTP, 1 mM GTP, UTP); 2 μl 10 mM GpppG cap (Pharmacia); 2 μl a [32P] -UTP (NEN) 800 Ci/mmol; 0.2 μl RNasin (Promega); 1 μl 0.1M DTT; 1.8 μl H2O; 0.5 μl Linearized Transcription Template (1 μg/μl); 0.5 μl Polymerase (SP6/T7/T3). After a 1-h incubation at 37°C. About 10 μl of the STOP solution (formamide loading buffer) was added for each reaction, boiled, and loaded onto a pre-run 5% denaturing polyacrylamide gel. Run until the desired distance. Cut out bands and soak in 500 μl RNA elution buffer (300 mM NaOAc, pH 6.1, 0.2% SDS, 1 mM EDTA) for 1 h overnight. Precipitate RNA with two volumes of ethanol. Resuspend in 20 μl of H_2_O and quantitate 0.5 μl.

RNA is bound to streptavidin magnetic beads. Add 50 μl of streptavidin magnetic beads to a 1.5 ml EP tube. Place the EP tube into a magnetic stand and aspirate the liquid. Add 50 μl of 20 mM Tris, pH 7.5 and resuspend. Magnetic beads; place the EP tube into a magnetic stand and aspirate the liquid; add 50 μl of 1 × RNA Capture Buffer to resuspend the magnetic beads; add a 50 pmol RNA probe to the magnetic beads and mix; incubate at room temperature for 30 min. The protein binds to RNA. Add 50 μl of streptavidin magnetic beads to a 1.5 ml EP tube. Place the EP tube in a magnetic stand and aspirate the liquid. Add 50 μl of 20 mM Tris, pH 7.5 to resuspend the magnetic beads. Put in a magnetic stand and aspirate the liquid; add 100 μl of 1 × Protein-RNA Binding Buffer to the magnetic beads and mix well; prepare a Protein-RNA Binding Reaction Master Mix; place the EP tube into the magnetic stand and aspirate the liquid. Add 100 μl Master Mix and mix; incubate at 4°C for 60 min. Elute the RNA-Binding protein, put the EP tube into a magnetic stand, and aspirate the liquid; add 100 μl of 1 × wash buffer, mix well, put the EP tube into the magnetic stand, and aspirate the liquid; add 50 μl Elution buffer, mix incubate at 37°C for 30 min. Place the EP tube into a magnetic stand, collect the liquid, and store at −20°C for Western blot or mass spectrometry.

### RNA extraction and quantitative real-time (qRT)-PCR

Cultured cells were collected to isolate total RNA through Trizol (Invitrogen) according to the manufacturer’s protocol. Total RNA from the cell lines was purified with the RNeasy Mini Kit (QIAGEN). RNA reverse transcription into cDNA was carried out with a Reverse Transcription cDNA Kit (Thermo Fisher Scientific, Waltham, U.S.A.). qPCR experiment was conducted with SYBR Green PCR Master Mix (Roche, Basle, Switzerland) on opticon RT-PCR Detection System (ABI 7500, Life Technology, U.S.A.). The expression levels of the above genes were analyzed by the 2^−ΔΔCT^. GAPDH expression was used for normalization. Divergent primers to detect circGOLPH3 were designed for PCR products of sizes ranging from 100 to 150 bp and spanning the junction site. The primer sequences were listed as follows: circGOLPH3, forward-GGTTACAACTAGAGGCTTGTGGA, reverse-CAGCCACGTAATCCAGATGAT-; CBX7, forward-5′-GCGTGCGGAAGGGTAAAGT-3′, reverse-5′-GCTTGGGTTTCGGACCTCTC-3′; GAPDH, forward-5′-AGCCACATCGCTCAGACACC-3′, reverse-5′-CGCCCAATACGACCAAATCC-3′.

### RNA-binding protein immunoprecipitation (RIP) assay

Cells were harvested when they reached 70–80% confluence. In brief, 2 × 10^7^ cells were washed in 4 ml ice-cold phosphate-buffered saline (PBS), centrifuged at 1000 rpm for 5 min and then lysed 1.7 ml polysome lysis buffer, 17 μl protease inhibitor, and 7.5 μl RNase inhibitor. The cell lysis sample was divided into IP, IgG, and Input, respectively. These samples were incubated with 5 µg anti-CBX7 antibody or negative control IgG (Abcam, U.K.) at 4°C for 2 h. A total of 40 µl of 50% slurry of protein A-Sepharose (GE Healthcare, Chicago, U.S.A.) was added to each sample, and the mixtures were incubated at 4°C for 4 h. The pellets were washed with 3× PBS and resuspended in 0.5 ml Tri Reagent (Sigma-Aldrich). The coprecipitated RNA eluted in aqueous solution was analyzed by qRT-PCR to prove the presence of binding products.

### Statistical methods

Each sample was testified in triplicate, and the results were expressed as the mean ± standard deviation (SD). An independent sample *t*-test was used for the analysis of the differences between the two groups. *P*<0.05 was considered statistically significant.

## Result

### Cell identification

The expressions of CD133, CD44, and Integrin alpha2beta1 in PC-3 cells were detected by immunofluorescence. Co-expressed CD133, CD44 and alpha2beta1 intergrin have been used as a marker to identify prostate cancer stromal cells previously as described by Ruan et al., 2019 [7]. The results showed that PC-3 cells were positive for CD133, CD44, Integrin alpha2beta1, and cell purity was considerable (Figure 1A). The qRT-PCR assay was used to detect the expression of circGOLPH3 in PC-3 and RWPE-1. The results showed that circGOLPH3 was significantly overexpressed in PC-3 cell lines (Figure 1B).

**Figure 1:** The identification of PC-3 cells by immunofluorescence (**A**) Immunofluorescence identification of CD133, CD44, Integrin alpha2beta1 expression in PC-3. (**B**) qPCR detection of circGOLPH3 expression in PC-3 and RWPE-1 cells. Data represent the average of three experiments and error bars indicate SD. Student’s *t*-test was used for the analysis of the differences between the two groups. ** indicated *P*<0.01.

### The circGOLPH3 promotes prostate cancer proliferation

CircGOLPH3 was overexpressed or interfered in cultured prostate cancer cells PC-3, and the cell cycle was detected by flow cytometry. The percentages of S-phase cells in the circGOLPH3-overexpressed group, overexpression control, the interference, and interference control were 61.26%, 42.56%, 30.52%, and 53.55% (Figure 2A), respectively. The Edu positive rates of the four groups’ cells were 85.65%, 20.26%, 4.65%, and 26.56%, respectively (Figure 2B). Overexpression of circGOLPH3 significantly increased the S-phase and Edu positive PC-3 cells, whereas silencing circGOLPH3 showed the opposite effect.

**Figure 2:** The circGOLPH3 promotes prostate cancer cell PC-3 proliferation (**A**) Cell cycle detection by flow cytometry. Bar graph shows the percentage of S phase cells. (**B**) Cell proliferation was detected by Edu staining. Bar graph shows the percentage of Edu positives cells. (**C**) Detection of cell viability by CCK8 Kit. (**D**) Detection of cell growth by MTT assay. OE indicated gene overexpression, si indicated gene silencing, and NC indicated negative control. Each bar was testified in triplicate, and data were expressed as the mean ± SD. Student’s *t* test was used for the analysis of the differences between the two groups. * indicated *P*<0.05; ** indicated *P*<0.01.

CCK8 Kit was used to detect cell proliferation activity. Proliferative activities of the four groups were 162%, 100%, 88%, and 99%, respectively (Figure 2C). Results of MTT assay reflected cell growth of the four groups, and the cell growth rates of the four groups were 158%, 100%, 65%, and 102% in respective (Figure 2D). There were statistically significant effects between the overexpression circGOLPH3 and overexpression control group, as well as silencing circGOLPH3. All results above indicated that overexpression of circGOLPH3 promoted the proliferation of PC-3 cells, and the interference circGOLPH3 efficiently reduced the proliferative activity of PC-3 cells.

### CircGOLPH3 inhibits apoptosis of prostate cancer cells

Apoptosis rates of the PC-3 cells were estimated by flow cytometry after the separate overexpression and interference to circGOLPH3. And results showed that the respective percentage of Annexin +/PI- cells in the overexpression, the overexpression control, the interference, and the interference control are 12.01%, 18.28%, 36.43%, and 17.57% (Figure 3A). The positive rates of TUNEL in the four groups of cells were 6.0%, 10.5%, 12.3%, and 10.0% in several (Figure 3B). The results of flow cytometry and TUNEL assays were statistically significant effects between the transfection and control groups. The above results indicate that over-expression of circGOLPH3 inhibits apoptosis of prostate cancer cells, and that interference with circGOLPH3 increases apoptosis rate of prostate cells.

**Figure 3:** The circGOLPH3 inhibits prostate cancer cell apoptosis (**A**) Apoptosis was detected by flow cytometry. (**B**) TUNEL staining to detect the cell apoptosis, bar graph shows the positive cell of TUNEL. Data represent the average of three experiments and error bars indicate SD. OE indicated gene overexpression, si indicated gene silencing, and NC indicated negative control. Student’s *t* test was used for the analysis of the differences between the two groups. * indicated *P*<0.05, ** indicated *P*<0.01.

### There is a binding effect of circGOLPH3 and CBX7 in their interaction

CircGOLPH3 was obtained through *in vitro* transcription, which was incubated with total protein from prostate cancer cells. The protein bound to circGOLPH3 was identified by RNA-pulldown and mass spectrometry (Figure 4A,B). Based on the mass spectrometry results, we found that CBX7 could specifically bind to circGOLPH3 and that the CBX7 was highly expressed in PC-3 cells (Figure 4C). To further verify the interaction between CBX7 and circGOLPH3, RNA immunoprecipitation (RIP) of CBX7 was performed in PC-3 cells, and then the expression of circGOLPH3 was analyzed by qRT-PCR. The results showed that CBX7 specific antibodies could precipitate CBX7 protein from cell lysates (Figure 4D), and circGOLPH3 was highly enriched in CBX7 immunoprecipitation particles when compared with the control (Figure 4E).

**Figure 4:** CircGOLPH3 binds to CBX7 (**A**) Silver pulldown detects RNA pulldown products; mass spectrometry detects RNA pulldown products. (**B**) The results of mass spectrometry for transcription of circGOLPH3 in vitro. (**C**) qPCR detects CBX7 expression in prostate cancer cells and 293-T cells. (**D**) CBX7 was measured by RIP assay. (**E**) CBX7 RIP assay of circGOLPH3 in PC-3 cells. circHIPK3 expression was detected by qRT-PCR. Data represent the average of three experiments and error bars indicate SD. Student’s *t* test was used for the analysis of the differences between the two groups. ** indicated *P*<0.01.

### Research on the regulation of CBX7 to the proliferation and apoptosis of prostate cancer cells

The vectors for CBX7 overexpression and interference were constructed, and respectively transfected into PC3 cells, and then the cell cycles were detected by flow cytometry. The percentages of S phase cells in the overexpression, overexpression control, interference, and interference control groups were 52.51%, 37.04%, 31.28%, and 44.98% in several (Figure 5A,B). CCK8 was performed to measure cell proliferation activity. The cell proliferation activities of the four groups were 188%, 100%, 71%, and 101%, respectively (Figure 5C). Results of MTT displayed the cell growth of the four groups were 169%, 100%, 52%, and 101%, respectively (Figure 5D). Apoptosis rate assay showed that the percentages of Annexin +/PI- cells in the four groups were 7.79%, 21.42%, 48.84%, and 23.43%, respectively (Figure 6A). The positive rates of TUNEL in the four groups of cells were 7.5%, 10.2%, 13.9%, and 10.9%, respectively (Figure 6B). The above results showed that CBX7 overexpression markedly promoted cell proliferation and reduced apoptosis, while the reverse was the case for circGOLPH3 silencing. Given that, CBX7 functions alike as circGOLPH3, which promotes proliferation and inhibits the apoptosis of prostate cancer cells.

**Figure 5:** CBX7 regulates the proliferation of prostate cancer cells PC-3 (**A** and **B**) Cell cycle detection by flow cytometry. (**C**) Detection of cell viability by CCK8. (**D**) Detection of cell growth by MTT. Data represent the average of three experiments and error bars indicate SD. Student's t test was used for the analysis of the differences between the two groups. ** indicated *P*<0.01.

**Figure 6:** CBX7 regulates the apoptosis of prostate cancer cells PC-3 (**A**) The apoptosis detection by flow cytometry. (**B**) The apoptosis detection by TUNEL staining. Data represent the average of three experiments and error bars indicate SD. Student's t test was used for the analysis of the differences between the two groups. * indicated *P*<0.05. ** indicated *P*<0.01.

## Discussion

Earlier clinical symptoms of prostate cancer patients are not obvious enough. However, once the clinical manifestations come to be, a local infiltration or a distant metastasis might have occurred. The 5-year survival rate of the local primary prostate cancer reaches almost 100% [1,2]; nevertheless, the 5-year survival rate of prostate cancer is only 28%. The occurrence and the development of prostate cancer are closely related to the tumor microenvironment. The composition of tumor microenvironment includes tumor cells, fibroblasts, myofibroblasts, immune cells, and the active media secreted by the cells, as well as blood vessels and/or lymphatic vessels, extracellular matrix, and so on [3,5]. The expression level of circHIPK3 is signally up-regulated in many tumor tissues such as prostate and renal cell carcinoma. In prostate cancer, circCSNK1G3 promotes cell proliferation by interacting with miR-181. Analysis of transcriptome data shows that after circCSNK1G3 is knocked out, cell cycle-related genes turn highly enriched. In human prostate cancer cell PC-3, miR-181b/d overexpression remarkably reduces the abundance of the tumor suppressor CBX7 [8]. Overexpression of miR-181b/d induces up-regulation of the cyclins CDK1 and CDC25A. However, knockout of circCSNK1G3 down-regulates both the expressions of CDK1 and CDC25A. Additionally, overexpression of miR-181b/d promotes PC-3 cell proliferation [8]. circ-SMARCA5 is an oncogene for prostate cancer, which promotes cell cycle and inhibits apoptosis [9].

Unlike linear RNA, the structure of circRNA is a covalently closed loop with no tail at the 5′-3′ port. This structure is endowed with the resistance against digestion of RNase that keeps itself intact. Therefore, circRNA is an ideal candidate for tumor diagnosis, monitoring, and prognosis [6,10]. CircRNAs are new members of non-coding RNAs. They are single-stranded closed-loop RNA molecules that exist in the body and are mainly produced by exon or intron sequences. Studies have found that circRNAs are widely involved in the regulation of many important life activities such as cell proliferation, differentiation, and apoptosis in vivo. CircRNAs have been researched in-depth in tumorigenesis mechanism, diagnosis and treatment, and these researches made some progress [11,12]. Scientists discovered that circRNAs participate in the regulation of biological processes by competitively binding miRNAs, interacting with RNA-binding proteins, maintaining the stability of mRNAs as well as regulating gene transcription, and participating in protein translation. Moreover, previous studies showed that circRNAs are closely related to many diseases such as neurological degenerative diseases, cardiovascular system diseases, diabetes, and tumors. Differentially expressed in the occurrence and development of digestive system common cancers. CircRNAs are involved in various biological processes of tumor cells [13–15]. CircRNAs sometimes function as miRNA sponges to promote tumor proliferation and invasion. They also affect the formation and development of tumors through the interaction with miRNAs. And they also inhibit the growth, proliferation, invasion and migration of tumor cells through different signaling pathways’ occurrence and development. In recent years, some scholars proposed a competitive endogenous RNA hypothesis. They believe that the RNA molecules with the same miRNA response element (MRE) competitively bind the same miRNA to achieve pairing targeted miRNA regulation. CircRNAs, also discovered as a newly important member of the ceRNA family, are rich in miRNA-binding sites. It serves as a ‘sponge effect’ to adsorb miRNA, reducing the inhibitory effect of miRNA on target genes and increasing the expression level of target genes, thus regulating biological processes. RNA-binding protein (RBP) acts as an activator or inhibitor of circRNA formation [16] which affects precursor mRNA formation, mRNA conversion, and translation, etc., and plays a role in a variety of cancers and other diseases. *In vitro* experiments with cell line models have found that f-circRNA activates the PI3K and MAPK signal transduction pathways, and it promotes primitive carcinogenesis and proliferation amid cancer development. Chromosomal translocations that occur during tumor cell replication produces abnormal fusion-circRNA (f-circRNA) [17]. An oncogenic fusion protein is formed by joining two separate genes together, leading to the formation of a fusion gene and the production of a mutant protein. This fusion protein makes cancer develop and progress. Circ-Foxo3 is capable of binding many types of proteins. It interacts with cyclin-dependent protein kinase 2 (CDK2) and other factors, thereby stopping the cell proliferation cycle in the G1/S phase [18].

Bachmayr-Heyda et al. studied the cancer tissues and adjacent tissues of patients with colon cancer and found that most of the relevant circRNAs were down-regulated. Five kinds of circRNAs are randomly selected for confirmation experiments, of which four were down-regulated. Similarly, compared with normal colon tissue, cirITCH expression is also down-regulated in colon cancer tissues. CirITCH increases the expression level of ITCH with its miRNA sponge function, while ITCH gene is involved in the Wnt/β-catenin pathway that is related to the pathogenesis of colon cancer related to progress; hence, this suggests that cirITCH may become a new marker candidate for the diagnosis of colon cancer. cir-cRNA_100876 is related to lymph node metastasis and staging of lung cancer. In bladder cancer tissues, the expressions of circFAM169A and circTRIM24 are up-regulated, while the other four are down-regulated, namely circTCF25, circZFR, circPTK2, and circBC048201. Recent studies have shown that circHIAT1 the metastasis inhibitor inhibits the migration and invasion of androgen receptor-enhanced renal cell as well as carcinoma cell, and it also increases the expression of circHIAT1 to target androgen receptor inhibition, thereby inhibiting the invasion and migration capabilities of renal cell carcinoma [19,20].

In colorectal cancer, hsa-circ-001569 up-regulates its downstream target genes E2F5, BAG4 and FMNL2 by adsorbing miR-145 to promote the proliferation and invasion of colorectal cancer tumor cells [21]. In the present study, after circGOLPH3 was overexpressed in prostate cancer cell line PC-3, and the proliferation and the cell viability of prostate cancer cells are greatly increased, and apoptosis is inhibited [22]. Moreover, the interference in circGOLPH3 reduces the proliferation of prostate cancer cells PC-3 as well as the cellular viability; and reversely, apoptosis was promoted. CircGOLPH3 binding protein was identified by mass spectrometry. At the same time, the CBX7 protein was highly expressed in prostate cancer cells, which was screened according to TCGA database comparison results. CBX7 function tests found that after overexpressing CBX7, the proliferative capacity and the cell viability of prostate cancer cells also robustly increased while apoptosis decreasing, consistent with the results of circGOLPH3 overexpression; after CBX7 expression interfered, the prostate cancer cell proliferation activity decreased and the apoptosis was increased. Our study demonstrated that circGOLPH3 and its binding protein circGOLPH3 promote proliferation and inhibit apoptosis in the prostate cancer cell.

## Abbreviations

CDK2: cyclin-dependent protein kinase 2
MRE: miRNA response element
PBS: phosphate-buffered saline
RBP: RNA-binding protein
RIP: RNA-binding protein immunoprecipitation
